This article has been retracted.

# CircPSMC3 suppresses the proliferation and metastasis of gastric cancer by acting as a competitive endogenous RNA through sponging miR-296-5p

**DOI:** 10.1186/s12943-019-0958-6

**Published:** 2019-02-18

**Authors:** Dawei Rong, Chen Lu, Betty Zhang, Kai Fu, Shuli Zhao, Weiwei Tang, Hongyong Cao

**Affiliations:** 1 Department of General Surgery, Nanjing First Hospital, Nanjing Medical University, Nanjing, Jiangsu China; 2 Michael G. DeGroote School of Medicine, McMaster University, Hamilton, Ontario Canada; 3 Department of General Clinical Research Center, Nanjing First Hospital, Nanjing Medical University, Nanjing, Jiangsu China

**Keywords:** Gastric cancer, circPSMC3, miR-296-5p, PTEN, Therapy

## Abstract

**Background:**

Circular RNAs (circRNAs) are a class of non-coding RNAs with a loop structure, but its functions remain largely unknown. Growing evidence has revealed that circRNAs play a striking role as functional RNAs in the progression of malignant disease. However, the precise role of circRNAs in gastric cancer (GC) remains unclear.

**Methods:**

CircRNAs were determined by human circRNA array analysis and quantitative reverse transcription polymerase reaction. Luciferase reporter, RNA pull down, and fluorescence in situ hybridization assays were employed to test the interaction between circPSMC3 and miR-296-5p. Ectopic over-expression and siRNA-mediated knockdown of circPSMC3, proliferation, migration and invasion in vitro, and in vivo experiment of metastasis were used to evaluate the function of circPSMC3.

**Results:**

CircPSMC3 rather than liner PSMC3 mRNA was down-regulated in GC tissues, corresponding plasmas from GC patients as well as GC cell lines compared to normal controls. Lower circPSMC3 expression in GC patients was correlated with higher TNM stage and shorter overall survival. Over-expression of circPSMC3 and miR-296-5p inhibitor could inhibit the tumorigenesis of gastric cancer cells in vivo and vitro whereas co-transfection of circPSMC3 and miRNA-296-5p could counteract this effect. Importantly, we demonstrated that circPSMC3 could act as a sponge of miR-296-5p to regulate the expression of Phosphatase and Tensin Homolog (PTEN), and further suppress the tumorigenesis of gastric cancer cells.

**Conclusion:**

Our study reveals that circPSMC3 can serve as a novel potential circulating biomarker for detection of GC. CircPSMC3 participates in progression of gastric cancer by sponging miRNA-296-5p with PTEN, providing a new insight into the treatment of gastric cancer.

**Electronic supplementary material:**

The online version of this article (10.1186/s12943-019-0958-6) contains supplementary material, which is available to authorized users.

## Introduction

Gastric cancer (GC) is the fifth most common cancer in the world and the third most common cause of cancer death worldwide [1]. It tends to metastasize into neighboring tissues and organs through lymph nodes and generate more cancer cells through the blood [2]. Although there have been many advancements in the diagnosis and treatment of GC, recurrence and metastasis are still occurring at high rates [3, 4]. Improvements in clinical care for these patients are limited by the lack of clarity surrounding the molecular mechanism in GC development [5]. Thus, it is urgently necessary to explore new potential biomarkers and their molecular mechanisms to better understand the pathophysiology of gastric malignancies.

Circular RNAs (circRNAs) are a new class of endogenous non-coding RNAs characterized by covalently closed loops without 5′ to 3′ polar or polyadenylation tails [6]. Previous studies have shown that circRNAs are formed by the back-splicing of pre-mRNA transcripts from genes with five different forms [7]. CircRNAs are stable, conserved and abundant in various cancer tissues or cell lines, as tissue/developmental stage-specific circRNAs are usually notable [8, 9]. Kuei-Yang Hsiao et al. found that circRNA CCDC66 could promote the progression and metastasis of colon cancer [10]. Studies on the molecular mechanism of circRNAs indicate that circRNAs can act as a competitive endogenous RNA (ceRNA) to regulate downstream genes associated with diseases by binding to miRNAs [11–13]. Xuetao Cao et al. found that circMTO1 might regulate the progression of hepatocellular carcinoma (HCC) by regulating the expression of p21 as a sponge of oncogenic miR-9, which can be used as a potential target for HCC therapy and a prognostic indicator for low patient survival [14]. Zhenyu Zhong et al. indicated that circMYLK could act as ceRNA of miR-29a, further promoting the progression of Epithelial-Mesenchymal Transition (EMT) in bladder cancer by activating VEGFA/VEGFR2 and Ras/ERK signaling pathways [15].

MicroRNAs (miRNAs), as a conserved small regulatory non-coding RNA, have been demonstrated to involve many biological functions in different diseases [16]. Many studies have reported that miRNAs can regulate by different circRNAs and lncRNAs to further regulate gene expression [17–19]. Yawei Li et al. found that circHIPK3, which contains two key binding sites of miR-558, directly regulates miR-558 function to inhibit heparanase (HPSE) expression. Their findings suggest that circHIPK3 acts as a “miRNA sponge” and identifies circHIPK3 as a new therapeutic target for patients with bladder cancer [20].

In this study, based on the results of circRNA arrays, we identified a circular RNA termed circPSMC3 derived from PSMC3 gene. CircPSMC3 was down-regulated in tissues, corresponding plasmas from GC patients as well as GC cell lines and could act as a sponge of miRNA-296-5p to regulate the expression of Phosphatase and Tensin Homolog (PTEN), and further suppress the tumorigenesis of GC cells. Our findings provide insight into the treatment of gastric cancer and reveal a novel potential circulating biomarker for detection of GC.

## Materials and methods

### Cell cultures and patient tissues

Human gastric cancer cell lines (BGC823, MGC803, SGC7901, AGS, and MKN45) were purchased from Shanghai Institutes for Biological Sciences, China. The human gastric epithelial cell line GES-1 was obtained from the Cancer Institute and Hospital of the Chinese Academy of Medical Sciences (Beijing, China). All cell lines were cultured in RPMI 1640 medium (Gibco, Carlsbad, CA, USA) supplemented with 10% fetal bovine serum (Gibco, Vienna, Austria) and in a humidified incubator containing 5% CO_2_ at 37 °C.

One hundred and-six samples of GC tissues were matched to adjacent normal tissues and 10 ml preoperative blood venous blood were collected from the GC patients treated in Department of General Surgery, Nanjing Hospital, Nanjing Medical University during 2013 to 2016 in accordance with the Helsinki Declaration. Twenty-one samples of 10 ml normal venous blood were randomly obtained from the 50–90 years old individuals without any underlying diseases in physical examination center of Nanjing Hospital during 2015 to 2016. All these specimens were frozen in liquid nitrogen and stably stored at − 80 °C until RNA extraction. Histological and pathological diagnoses of these specimens were confirmed and classified by two experienced clinical pathologists. Informed consent from these patients has been obtained before specimen collection. This project was approved by the Ethics Committee of Nanjing Medical University.

### Quantitative reverse transcription polymerase reaction (qRT-PCR)

According to the manufacturer’s protocol, total RNAs from tissues, plasma and cells were isolated by using TRIzol reagent (Invitrogen, CA, USA). For circRNA and mRNA, cDNA was synthesized by using reverse transcription kit (Takara, Otsu, Japan) and for miRNA, total RNAs were reversed using RiboBio reverse transcription kit (Guangzhou, China). Quantification of mRNA and circular RNA was performed by using a SYBR Green PCR Kit (Takara, Otsu, Japan), and miRNA PCR was performed by using a SYBR Green PCR Kit (RiboBio,Guangzhou, China). All primer sequences were designed and synthesized by Genery (Nanjing, China). CircPSMC3 expression level was detected using the following primer pair: 5′-GTTTAGGGTCCCTGCCCTTTG-3′ (Forward, or F) and 5′-GTGTTGGGCTGGAAGCCATC-3′ (Reverse, or R). The primer pair of PSMC3 is 5′- AGACGCTGCCCACAGAGTATG -3′ (F) and 5′- CTTTTGGAGGTTGGATCCCC-3′ (R). GAPDH was used to normalize the mRNA and circRNA expression levels and U6 was used to normalize the miRNA expression levels before calculation.

### RNase R treatment

Total RNA (10 μg) of gastric cancer cell lines was mixed with 40 U RNase R at 37 °C for 2 h. To assess the stability of circPSMC3 and line PSMC3 mRNA, the expression levels were determined by using qRT-PCR.

### Oligonucleotide transfection

Si-circPSMC3, miRNA-296-5p mimic, miRNA-296-5p inhibitor and their related control oligonucleotide were designed and synthesized by RiboBio (Guangzhou, China). The sequence of siRNA:siRNA-1:TAGGGTCCCTGCCCTTTGA, siRNA-2:GGGTCCCTGCCCTTTGACA, siRNA-3: TCCCTGCCCTTTGACAGTG. All transfections were performed by the final concentration of 60 nM of miRNA mimics and 100 nM of miRNA inhibitor and si-circPSMC3. Lipofectamine 2000 reagent (Invitrogen) was used as transfection medium.

### Plasmids construction and stable transfection

To isolate stable human gastric cancer cells over-expressing circPSMC3, circPSMC3 cDNA was synthesized cloned into pcD-ciR and pcDNA3 vector and lentivirus (Hanheng, Shanghai, China). According to the manufacturer’s instructions, human gastric cancer cell lines, MGC803 and BGC823 were infected with lentivirus at a multiplicity of infection of 50. All cell lines were followed by selection with 2 μg/mL puromycin for 2 weeks.

### Luciferase reporter assay

The wild-type and mutant fragments in 3′-UTR of circPSMC3 related with miRNA-296-5p binding site were designed, synthesized and inserted into pGL3-basic vectors (Realgene, Nanjing, China), then pGL3-basic vectors and miRNA-296-5p mimics or inhibitor or circPSMC3 overexpressing lentivirus were co-transfected to 293 T cell respectively. After 48 h, according to the manufacturer’s instructions, luciferase activity in co-transfected cells were collected and detected by the dual-luciferase reporter assay system (Promega).

### Biotin-coupled probe RNA pull down assay

Biotin-coupled probe RNA pull down assay was performed. To pull down the miRNA by circRNA, MGC803 and BGC823 with transfected with miRNA-296-5p mimics were lysed and incubated with Biotin-coupled probe of circPSMC3 which was pre-bound on magnetic beads. For 2 h, target RNA was pulled by the RNeasy Mini Kit (QIAGEN, Germany). Then the pull-down product was extracted, reversed and placed through q-PCR. To pull down the circRNA by miRNA, MGC803 and BGC823 with circPSMC3 over-expression and Biotin-coupled probe of miRNA-296-5p were processed through the same protocol.

### Fluorescence in situ hybridization (FISH)

The fluorescence in situ hybridization assay was performed to detect the presence of circPSMC3 and miRNA-296-5p by using Fluorescence in Situ Hybridization Kit (RiboBio, Guangzhou, China). CircPSMC3 was captured with Cy5-labeled probe and miRNA-296-5p was captured with Cy3-labeled probe respectively. After prehybridization, circPSMC3 probe and miRNA-296-5p probe were hybridized in prepared hybridization buffer in MGC803 cells. Nuclei were marked by staining with 4,6-diamidino-2-phenylindole (DAPI). Confocal microscopy was used to better visualize the presence of circPSMC3 and miRNA-296-5p.

### Cell counting kit-8 proliferation assay and 5-Ethynyl-20-deoxyuridine (EdU) incorporation assay

GC cells were seeded in 96 wells with the density of 4000 cells per well. Seeded cells were treated with 10 μl of CCK8 solution (Ribobio, Guangzhou, China) after cultured at 0 h, 24 h, 48 h, 72 h, 96 h, respectively. Then the absorbance of cells at each time was analyzed at 450 nM by microplate reader according to the manufacturer’s instructions (Synergy4; BioTek, Winooski, VT, USA). The EdU assay was performed to assess the proliferation of cells by using a Cell-Light EdU DNA Cell Proliferation Kit (RiboBio, Guangzhou, China). GC cells were plated in 24 wells and were cultured for 24 h. These two cell lines were fixed using 4% paraformaldehyde after incubation with 50 mM EdU solution for 2 h. Then according to the manufacturer’s protocol, cell lines were sealed with Apollo Dye Solution and Hoechst 33342 in order. The EdU cell lines were photographed and counted under an Olympus FSX100 microscope (Olympus, Tokyo, Japan).

### Transwell migration and invasion assays

For this assay, according to the manufacturer’s protocol, GC cells were seeded in upper chambers with 200 μl of serum-free medium. The transwell chamber (Corning, NY, USA) was paved with matrigel mix (BD Biosciences, San Jose, CA, USA) for invasion assays and without matrigel mix for migration assays. The bottom chamber was filled with medium and 10% FBS as a gastric cancer cell chemoattractant. After incubation for 24 h, the upper chambers were fixed and then stained by crystal violet (Kaigen, Nanjing, China) for 15 min. For visualization, the cell lines were photographed and counted in different five fields.

### Cell apoptosis assays

GC cells were stained with FITC and PI from the Annexin V-FITC/Propidium Iodide (PI) Apoptosis Detection Kit (BD Biosciences #556547). FACScan (BD Biosciences, San Jose, CA, USA) was used to analysis stained cells and all apoptosis data of different cell lines was analyzed by Flowjo V10 software (Tree Star, San Francisco, CA, USA).

### Western blot

Cells were lysed in RIPA lysis buffer (RIPA, Beyotime, China). The protein was prepared and quantified by bicinchoninic acid (BCA) analysis (Beyotime, China). The same amounts of protein were extracted by 10% SDS-PAGE and transferred onto a PVDF membrane (Millipore, Schwalbach, Germany). The blocked protein with 5% skim milk powder was incubated with primary antibody anti-PTEN (#3285, Cell Signaling Technology), anti-YYM (#66281–1-Ig, Proteintech), anti-GAPDH (#ab181602, Abcam).at 4 °C for 12 h.Then the prepared membranes were incubated with secondary antibody (1:5000) for 2 h. Finally, the blots were detected by enhanced chemiluminescence kit (Pierce, Waltham, MA, USA) and related data was analyzed by Image Lab Software.

### Xenografts in mice

The animal assay was approved by the animal management committee of Nanjing Medical University, and all experimental procedures and animal care were in accordance with the institutional ethics guidelines for animal experiments. To create the xenograft tumor model, 20 5-week-old male nude mice were separated randomly into over-circPSMC3 group and NC group (*n* = 10 for each group). About 1× 10^7^ circPSMC3 over-expressing MGC803 cells were subcutaneously injected into the axilla of the nude mice respectively. The volume of all injected nude mice was measured every 3 days by using digital calipers. After 35 days, all injected nude mice were sacrificed, excised tumor weights were measured and tumor tissues were studied by hematoxylin and eosin (H&E) and IHC staining. To produce the nude mice metastasis model, 20 5-week-old male nude mice were separated randomly into over-circPSMC3 group and NC group (*n* = 10 for each group). About 2× 10^6^ circPSMC3 over-expressing MGC803 cells were tail-vein injected into 20 5-week-old male BALB/c nude mice respectively. Six weeks later, the nude mice were sacrificed; pulmonary metastases nodules were counted by three pathologists after the lungs were removed by experienced surgeons. The lungs removed were studied by using hematoxylin-eosin staining.

### Statistical analysis

The analyses were mainly performed by using SPSS 19.0 (IBM, SPSS, and Chicago, IL, USA) and *p*-value < 0.05 was demarcated to be statistically significant. Comparison of continuous data was analyzed using an independent *t*-test between the two groups, whereas categorical data was analyzed by the chi-square test. Kaplan-Meier method was mainly used to assess the survival rate and analyzed by using log rank test.

## Results

### CircPSMC3 is significantly down regulated in gastric cancer and associated with poor prognosis

To investigate the role of circRNAs in the development of gastric cancer, the circRNA expression signatures in gastric cancer plasma were explored by using circRNA microarray analysis using plasma samples from 10 GC patients, including 5 patients with no lymph node metastasis and the other 5 patients with lymph node metastasis, and 5 normal individuals. The result showed that 6405 circRNAs in lymph node metastasis group and normal group (Fig. 1a) and 3443 circRNA in lymph node metastasis group and no lymph node metastasis group (Fig. 1b) were significantly altered with fold change > 2.0 and *P* < 0.05. GO pathway analysis suggest that these differentially expressed circRNAs are relevant to several vital physiological processes, molecular functions, and critical signaling pathways in two groups (Fig. 1c-d).

**Fig. 1:** CircPSMC3 expression is down regulated in clinical GC specimens and cell lines. **a** Scatter plot analyses of circRNAs microarray data showing differentially expressed circRNA in lymph node metastasis group and normal group . High expression level is indicated by “red” and low levels by “green”. **b** Scatter plot analyses of circRNA microarray data showing differentially expressed circRNAs in lymph node metastasis group and no lymph node metastasis group. **c** GO analysis of circRNAs in lymph node metastasis group and normal group. **d** GO analysis of circRNAs in lymph node metastasis group and no lymph node metastasis group. **e** The spliced mature sequence length of circPSMC3 derived from the PSMC3 gene is 502 bp. **f** QRT-PCR for the abundance of circPSMC3 in GC cells treated with RNase R. **g** QRT-PCR for the abundance of PSMC3 mRNA in GC cells treated with RNase R. **h** CircPSMC3 expressions were evaluated using qRT-PCR in 106 pairs of gastric cancer plasmas and 21 pairs of normal plasmas. **i** CircPSMC3 expressions were measured using qRT-PCR in 106 pairs of gastric cancer (Tumor) and matched noncancerous tissue (Normal). **j** The expressions of circPSMC3 were evaluated in cell lines using qRT-PCR. **k** The area under the ROC curve (AUC) in distinguishing GC plasmas and normal ones was 0.9326. **l** Kaplan Meier survival curve showed the relationship between circPSMC3 and survival rates. **p < 0.01, ***p < 0.001

We selected a total of 6 circRNAs based on the multiple fold difference in circRNA microarray and then verified the findings in a small sample of plasmas by using qRT-PCR as well as the structure, length, and source of circRNA (Additional file 1: Figure S1a). Results showed that a novel circRNA named circPSMC3, which has never been reported in previous literature, has a significantly lower expression in GC plasmas compared to normal controls, which was then picked out for further study. The spliced mature sequence length of circPSMC3 derived from the PSMC3 gene is 502 bp according to circbase database (http://www.circbase.org/) (Fig. 1e) and circPSMC3 is derived from exons, while no other subtypes of circPSMC3 are found. The stability of circPSMC3 was evaluated and results showed that circPSMC3 harbors a loop structure with the resistance to digestion by RNase R (Fig. 1f), while PSMC3 mRNA could be degraded by RNase R (Fig. 1g).

Given that the tremendous diagnostic and therapeutic role of circRNAs in GC, we explored the clinical value of circPSMC3 by detecting its expression in GC samples. Results indicated circPSMC3 had significantly lower expression in GC plasmas (Fig. 1h), tissues (Fig. 1i) and cells (Fig. 1j) compared to normal controls. In addition, circPSMC3 expression was lower in preoperative blood from GC patients with lymph node metastasis compared to those patients without lymph node metastasis (Fig. 1h). Clinicopathological features showed that down-expression of circPSMC3 was negatively associated with TNM stage (Table 1, *P* = 0.000) and lymphatic metastasis (Table 1, *P* = 0.021). However, circPSMC3wa not associated with the gender, age, size, or histological grade. Furthermore, the area under the ROC curve (AUC) of circPSMC3 in distinguishing GC plasmas and normal ones was 0.9326 (Fig. 1k) and the cut-off value was − 9.965 with the sensitivity of 85.85% and specificity of 95.24%. Kaplan-Meier overall survival curve revealed that patients with lower circPSMC3 expression showed a reduced overall survival time (Fig. 1l).

**Table 1:** Correlations between circPSMC3 expression in plasmas and clinical characteristics in GC patients

characteristic	case	circPSMC3 expression		*p* value
		low	high	
All cases	106	91	15	
Age (yeas)				0.530
< 65	40	34	6	
≥65	66	57	9	
Gender				0.250
Female	37	34	3	
Male	69	57	12	
Tumor size (cm)				0.266
< 5	42	34	8	
≥5	64	57	7	
Histological grade				0.309
High	23	18	5	
Middle-low	83	73	10	
Lymph node metastasis				0.021^*^
Negative	27	19	8	
Positive	78	72	7	
TNM stage				0.000^*^
I–II	38	24	14	
III–IV	68	67	1	

^*^indicates *P* < 0.05

### CircPSMC3 plays a suppression role in gastric cancer cells in vitro

To evaluate the role of circPSMC3 in GC cells, three siRNAs against circPSMC3 were designed to silence circPSMC3 without influencing PSMC3 mRNA level in BGC823 and SGC7901 cells (Additional file 1: Figure S1b-1d) and finally si-circPSMC3#1 was chosen for the following experiment with its high inhibitory efficiency. The circular transcript expression vector circPSMC3 was successfully constructed in MGC803 and AGS cells (Fig. 2a), as it could increase circPSMC3 expression level rather than PSMC3 mRNA (Additional file 1: Figure S1e-1f). The results of CCK-8 and EdU assay showed that si-circPSMC3 could promote cell proliferation in BGC823 and SGC7901 cell lines, whereas over-expression of circPSMC3 (named circ-PSMC3) might inhibit cell proliferation in MGC823 and AGS cell lines (Fig. 2b-c). Wound healing assay showed that silencing of circPSMC3 significantly increased the cell mobility, while over-expression of circPSMC3 might inhibit the cell mobility (Fig. 2d). The result of cell invasion assay showed that down regulation of circPSMC3 significantly increased cell invasion and over-expression of circPSMC3 exhibited the opposite role (Fig. 2e).

**Fig. 2:** CircPSMC3 produces suppression effects on gastric cancer cells. **a** The circular transcript expression vector circPSMC3 was constructed. **b** The growth curves of cells were measured after transfection with circPSMC3 vector or Mock vector or si-circ or si-NC by using CCK-8 assays. **c** EdU assays of GC cells transfected with control or circPSMC3 siRNAs or circPSMC3 vector or Mock were performed to evaluate cell proliferation. **d** Cell motility was examined in cells transfected with circPSMC3 vector or Mock vector or si-circ or si-NC by wound healing assay. **e** Cell invasion assays were performed in cells transfected with control or circPSMC3 siRNAs or circPSMC3 vector or Mock. Data indicate mean ± SD of at least three independent experiments. *p < 0.05, **p < 0.01, ***p < 0.001, Scale bar, 100 mm

### CircPSMC3 directly binds to miR-296-5p and suppresses miR-296-5p activity

Given that circRNAs could bind to different miRNAs and regulate downstream genes, we found that circPSMC3 possessed a complementary sequence to miR-296-5p seed region by bioinformatics analysis through Circinteractome database (https://circinteractome.nia.nih.gov/). To confirm the website prediction, the biotin-coupled probe pull-down assay was performed and the results showed miR-296-5p and circPSMC3 were detected in the circPSMC3 pulled-down pellet compared with the control group (Fig. 3a). Furthermore, the result of FISH indicated that circPSMC3 was co-localized with miR-296-5p in the cytoplasm of MGC803 cell lines (Fig. 3b).

**Fig. 3:** CircPSMC3 directly binds to miR-296-5p and suppresses miR-296-5p activity. **a** Lysates from MGC803 and AGS cells with circPSMC3 vector were subjected to biotinylation-cirPSMC3 pull down assay, and expression levels of circPSMC3 and miR-296-5p were measured by qRT-PCR. **b** The Schematic of circPSMC3 wild-type (WT) and mutant (Mut) luciferase reporter vectors. **c** The relative luciferase activities were analyzed in 293 T cells co-transfected with miR-296-5p mimics or miR-NC and luciferase reporter vectors psiCHECK2-circPSMC3-WT or psiCHECK2-circPSMC3-Mut. **d** The expressions of miR-296-5p were analyzed by using qRT-qPCR in cells transfected with circPSMC3 or mock vector or si-circ or si-NC vector. **e** The expression levels of circPSMC3 were determined with qRT-qPCR in cells transfected with miR-296-5p mimics or inhibitor. Data indicate mean ± SD, n ¼ 3. **P < 0.01, ***P < 0.001

In addition, luciferase reporters with either the wild type circPSMC3 sequence (WT) or the sequence with mutated binding sites of miR-296-5p (Mut) into the 3 UTR of renilla luciferase showed that miR-296-5p over-expression could significantly reduce the luciferase activities of WT reporter rather than mutant one (Fig. 3c). QRT-PCR further confirmed that circPSMC3 knockdown could increase the miR-296-5p level and circ-PSMC3 had an opposite role in GC cell lines (Fig. 3d). However, miR-296-5p failed to influence circPSMC3 level (Fig. 3e). Collectively, these revealed that circPSMC3 could bind to miR-296-5p to further regulate its expression level.

### MiR-296-5p targets PTEN and promotes the proliferation and invasion of gastric cancer cells

According to miRanda database prediction (http://mirdb.org/), miR-296-5p could target PTEN mRNA 3′ UTR with a high score.

This interaction was confirmed by performing luciferase reporter assays. The results showed that the over-expression of miR-296-5p could significantly reduce the activity of a luciferase reporter compared to miR-NC and the inhibition of the miR-296-5p may evidently increase the luciferase activity compared with inh-NC with wild type PTEN sequence (WT), however, these effect disappeared with mutated binding sites of miR-296-5p (Mut)(Fig. 4a). The knockdown or over-expression model of miR-296-5p was successfully established (Additional file 1: Figure S1g-1 h). We found that miR-296-5p over-expression significantly reduced the PTEN mRNA levels in GC cells (Fig. 4b). Western blot further confirmed that transfection of miR-296-5p mimics could reduce PTEN expression (Fig. 4c). These results showed that miR-296-5p could negatively regulate the expression of PTEN.

**Fig. 4:** MiR-296-5p can promote GC cell activities by targeting PTEN. **a** The Schematic of PTEN 3 UTR wild-type (WT) and mutant (Mut) luciferase reporter vector were shown. The relative luciferase activities were analyzed in 293 T cells co-transfected with miR-296-5p mimics or miR-NC or in-296-5p or in-NC. **b** The relative expressions of PTEN mRNA were evaluated by using qRT-qPCR in cells transfected with the miR-296-5p mimics or inhibitors respectively. **c** The relative expressions of PTEN protein were evaluated by using western blot in cells transfected with the miR-296-5p mimics. **d** The growth curves of cells were measured after transfection with miR-296-5p mimics or inhibitor by using CCK-8 assays. **e** EdU assays of GC cells transfected with miR-296-5p mimics or miR-NC were performed to evaluate cell proliferation. **f** Cell motility was examined in cells transfected with miR-296-5p mimics or miR-NC by wound healing assay. **g** Cell invasion or migration assays were performed in cells transfected with miR-296-5p mimics or miR-NC by using using transwell chamber with or without matrigel respectively. Data indicate mean ± SD of at least three independent experiments. *p < 0.05, **p < 0.01, ***p < 0.001, Scale bar, 100 mm

The role of miR-296-5p on the GC cell proliferation, viability, invasion, and migration was evaluated. The results indicated that over-expression of miR-296-5p promoted the proliferation (Fig. 4d-e), migration (Fig. 4f) and invasion (Fig. 4g) of GC cells. However, down expression of miR-296-5p might exert an opposite effect (Fig. 4d). These results suggest that miR-296-5p could target PTEN and further promote the development of GC partially.

### CircPSMC3 suppresses the proliferation and invasion of gastric cancer by sponging miR-296-5p to regulate PTEN

In order to further explore the interaction among circPSMC3, miR-296-5p and PTEN, we performed luciferase reporter assays. The data showed that the over-expression of circPSMC3 could significantly increase the activity of a luciferase reporter, however, the co-transfection of circPSMC3 and miR-296-5p may eliminate this effect with wild type PTEN sequence (WT), and these effects disappeared with mutated binding sites of miR-296-5p (Mut)(Fig. 5a). Moreover, we found that circ-PSMC3 significantly increased the PTEN mRNA levels, whereas co-transfection of circ-PSMC3 and miR-296-5p may cancel out this effect in MGC803 and AGS cells (Fig. 5b). Western blot showed that circ-PSMC3 could promote PTEN expression, while co-transfection of circ-PSMC3 and miR-296-5p had no effect on PTEN level (Fig. 5c). These results demonstrated that circPSMC3 could regulate PTEN expression by acting as a competing endogenous RNA to sponge miR-296-5p. Results of the malignant behavior of circPSMC3 and miR-296-5p on GC cell proliferation, viability, invasion migration and metastasis indicated that the circ-PSMC3 could inhibit proliferation, invasion and migration of GC cells. However, co-transfection of circPSMC3 and miR-296-5p may counteract this effect (Fig. 5d-h). These results of experiments suggested that CircPSMC3 suppresses the proliferation, invasion and migration of gastric cancer cells by sponging miR-296-5p to regulate PTEN.

**Fig. 5:** Over-expression of circPSMC3 regulates PTEN expression and inhibits GC cells activities by targeting miR-296-5p. **a** The relative luciferase activities were analyzed in 293 T cells co-transfected with circPSMC3 vector or Mock and miR-296-5p mimics or miR-NC and luciferase reporters vectors psiCHECK2- PTEN 3 UTR-WT or psiCHECK2-PTEN 3 UTR-Mut. **b** The expression levels of PTEN mRNA were analyzed using RT-qPCR in MGC803 and AGS cells were co-transfected withcircPSMC3 vector or Mock and miR-296-5p mimics or miR-NC. **c** The expression levels of PTEN protein were analyzed using Western blot in MGC803 and AGS cells were co-transfected with circPSMC3 vector or Mock and miR-296-5p mimics or miR-NC. **d** The growth curves of cells were measured after co-transfected with circPSMC3 and miR-296-5p mimics by using CCK-8 assays. **e** EdU assays of GC cells co-transfected with circPSMC3 and miR-296-5p mimics were performed to evaluate cell proliferation. **f** The cell apoptosis ability was evaluated by using apoptosis assay in cells co-transfected with circPSMC3 and miR-296-5p mimics. **g** Cell motility was examined in cells co-transfected with circPSMC3 and miR-296-5p mimics by wound healing assay. **h** Cell invasion or migration assays were performed in cells co-transfected with circPSMC3 and miR-296-5p mimics by using transwell chamber with or without matrigel respectively. Data indicate mean ± SD of at least three independent experiments. *p < 0.05, **p < 0.01, ***p < 0.001, Scale bar, 100 mm

### Circ-PSMC3 inhibits the growth and metastasis of gastric cancer in vivo

To explore the association between circPSMC3 and the growth as well as metastasis of gastric cancer in vivo, MGC803 cells transfected with circPSMC3 and GFP was injected into nude mice to established xenograft tumor model and metastasis nude mice model (Fig. 6a). In xenograft tumor model, we found that over expressing of circPSMC3 generated a negative effect on the volume of nude mice (Fig. 6b) as well as the weight (Fig. 6c). Ectopic over-expression of circPSMC3 inhibited metastasis in the lung compared to normal expression of circPSMC3 (Fig. 6d). Taken together, we illustrated that the over-expression of circPSMC3 could inhibit the proliferation, invasion and metastasis of GC cells and then suppress the progression of GC by sponging miR-296-5p to regulate PTEN expression (Fig. 6e).

**Fig. 6:** Over-expression of circPSMC3 inhibits the GC cells activities in vivo. **a** Representative images of the GC tumor bearing BALB/c nude mice and xenograft GC tumors. **b** The growth curves of xenograft tumors. The tumor volumes were measured every week. **c** The relative weights of tumors were evaluated. **d** The number of lung metastasis in over-expression of circPSMC3 and normal xenograft groups. **e** The schematic diagram of the mechanism of circPSMC3/miR-296-5p/PTEN axis in GC. **p < 0.01, ***p < 0.001

## Discussion

Deep sequencing combined with novel bioinformatics approaches led to the discovery that a significant portion of the human transcriptome is spliced into RNA loops [21]. In the last few years, several research groups have published interesting results, shedding light on the biogenesis of circRNAs and possible mechanisms involving them [22]. Some of these discoveries have shown that circRNAs are very stable, abundant and present a tissue-specific expression pattern [23].

In our study, we confirmed that circPSMC3 was significantly lower expressed in GC plasmas, tissues and cells compared to normal controls. Clinicopathological features illustrated that down expression of circPSMC3 was negatively associated with TNM stage and lymphatic metastasis, with a reduced overall survival time for GC patients. More and more studies have explored the relationship between circRNAs and the development of gastric cancer from a clinical perspective and investigated its application as a tumor biomarker in clinic. For example, Xie Y et al. detected the expression levels of hsa_circ_0074362 in 127 gastric cancer tissues and paired adjacent normal tissues by quantitative reverse transcription-polymerase chain reaction. Results showed hsa_circ_0074362 levels were significantly down regulated in gastric cancer tissues, gastritis tissues and gastric cancer cell lines and were associated with lymphatic metastasis, which may be a potential biomarker of gastric cancer [24]. However, most of the studies only detect the expression of circRNAs from cancer tissues and adjacent tissue. Only a small number of studies detect the expression of circRNAs from preoperative blood in GC patients and the sample size is small. The results of our study make circPSMC3 an ideal noninvasive biomarker for the diagnosis and prognosis of gastric cancer.

We demonstrated that miR-296-5p targets PTEN and promotes the proliferation and invasion of GC cells. Current studies show that miR-296-5p plays a role in cancers. For example, Lee H et al. observed that miR-296-5p promoted the invasion of various glioblastomas cells. From results obtained from Ago2 immunoprecipitation and luciferase assays, they found that miR-296-5p downregulated CASP8 and NGFR through direct interaction between seed sequence of the miRNA and 3’UTR of the target mRNA. Collectively, their results implicated miR-296-5p as a potential cause of invasiveness in cancer and identifies miR-296-5p as a promising therapeutic target for glioblastomas [25]. Maia D reported miR-296-5p expression is associated with resistance to radiotherapy and tumor recurrence in early stage laryngeal squamous cell carcinoma, showing the feasibility of this marker as a novel prognostic factor for this malignancy. Furthermore, miR-296-5p expression could be helpful in the identification of tumors resistant to radiotherapy, thus informing treatment plans [26]. Interestingly, Lee KH reported that miR-296-5p has a tumor-suppressive role by targeting Pin1. This suggested that there are likely prognostic and clinical applications of miR-296-5p in prostate cancer therapy [27]. In gastric cancer, Li T et al. showed miR-296-5p over-expression significantly promoted GC cell growth and attenuated the CDX1-induced anti-growth effects by recurring cell cycle distribution and apoptotic status, whereas knockdown of miR-296-5p decreased GC cell growth [28], which is consistent with our result.

There are accumulating examples of circRNAs acting as miRNA sponges, thereby influencing the posttranscriptional actions of miRNAs as suppressors of the translation and/or stability of target mRNAs [29, 30]. For example, cir-ITCH (Itchy E3 ubiquitin protein ligase) was reported to sponge miR-7, miR-17, and miR-214, leading to the upregulation of ITCH and the inhibition of WNT signaling in esophageal squamous cell carcinoma [31]. Li X found that hsa_circ_103809 could bind to miR-620 and negatively regulates miR-620 expression, further inhibiting the proliferation and invasion abilities of hepatocellular carcinoma cells [32]. In our research, we discovered that the over-expression of circPSMC3 could inhibit the proliferation, invasion and metastasis of GC cells. Furthermore, it can suppress the progression of GC by regulating miR-296-5p and PTEN expression. Functional inactivation of the tumor suppressor protein PTEN has been detected in multiple cases of GC, and already shown to be closely linked to the development, progression and prognosis of the disease. Inactivation of PTEN can be attributed to gene mutation, loss of heterozygosity, promoter hypermethylation, microRNA-mediated regulation of gene expression, and post-translational phosphorylation. PTEN is also involved in mechanisms regulating tumor resistance to chemotherapy [33]. Liu S et al. reported that low expression of PTEN and increased expression of miR-718 in GC tissues were both independent and unfavorable prognostic factors of GC. Up regulation of miR-718 could increase PI3K/Akt signaling by directly down regulating PTEN, thus promoting the proliferation and invasion of gastric cancer cells [34]. Liu T found that Circ-ZFR and PTEN were low-expressed whereas miR-107 and miR-130a were high-expressed in GC tissues and cells. There are targeted relationships and interactions between miR-130a/miR-107 and ZFR/PTEN. Circ-ZFR inhibits GC cell propagation, cell cycle and promoted apoptosis by sponging miR-107/miR-130a, while miR-107/miR-130a promoted GC cell propagation and prevented apoptosis through targeting PTEN. Circ-ZFR inhibited cell proliferation and facilitated apoptosis in GC by sponging miR-130a/miR-107 and modulating PTEN. Circ-ZFR curbed GC tumor growth and affected p53 protein expression in vivo [35]. To our knowledge, this is the first study to investigate the role of circPSMC3 in gastric cancer. Not only that, this is also the first article to study the relationship between miR-296-5p and PTEN. These findings may bring light to the treatment of GC.

There are several limitations to the interpretation of our study results. Firstly, our study uses GC samples taken from an ethnically homogenous population and expects further sample size and more validation from different regions. Secondly, our study examines the ability of circPSMC3 to bind to miR-296-5p, but there may be other miRNAs that binds circPSMC3 to regulate the occurrence and progression of GC. Thirdly, whether circPSMC3 regulates the development of GC through other mechanisms such as protein binding requires further investigation. We hope that a follow-up study will elucidate a deeper understanding of the therapeutic potential of circPSMC3.

## Conclusion

Our study identifies a new circular RNA, termed circPSMC3 that is down-regulated in tissues, corresponding plasmas from GC patients as well as GC cell lines and can act as a sponge of miRNA-296-5p to regulate the expression of PTEN. Our findings reveal a novel potential circulating biomarker for detection of GC.

## Additional file

Additional file 1: **Figure S1.** (a) A total of 6 circRNAs based on the multiple fold difference in circRNA microarray and then were verified in a small sample of plasmas by using qRT-PCR. (b) SiRNA against circPSMC3 were designed to silence circPSMC3 level in BGC823 cells. (c) SiRNA against circPSMC3 were designed to silence circPSMC3 level in SGC7901 cells. (d) SiRNA#1 against circPSMC3 were designed to silence circPSMC3 without influencing PSMC3 mRNA level in BGC823 and SGC7901cells. (e) The expression of circPSMC3 was evaluated in MGC803 and AGS cells transfected with circPSMC3 vector or Mock by using qRT-PCR. (f) The expression of PSMC3 mRNA was evaluated in MGC803 and AGS cells transfected with circPSMC3 vector or Mock by using qRT-PCR. (g) The expression of miR-296-5p was evaluated in MGC803 and AGS cells transfected with miR-296-5p inhibitor or miR-NC. (h) The expression of miR-296-5p was evaluated in MGC803 and AGS cells transfected with with miR-296-5p mimics or miR-NC. *p < 0.05, **p < 0.01, ***p < 0.001. (DOCX 722 kb)

## Abbreviations

CCK8: Cell counting kit-8
ceRNA: competitive endogenous RNA
circRNAs: Circular RNAs
EdU: 5-Ethynyl-20- deoxyuridine
GAPDH: Glyceraldehyde-3-phosphate dehydrogenase
GC: Gastric cancer
GO: Gene oncology
IgG: immunoglobulin G
KEGG: Kyoto Encyclopedia of Genes and Genomes
miRNAs: MicroRNAs
PTEN: Phosphatase and Tensin Homolog
qRT-PCR: Quantitative reverse transcription polymerase reaction
RIP: RNA immunoprecipitation
RNA-FISH: RNA fluorescence in situ hybridization
ROC: Receiver-operating characteristic
WT: Wild type
